# Design of Online Ideological and Political Teaching of Building Architecture from the Perspective of Machine Learning

**DOI:** 10.1155/2022/8347235

**Published:** 2022-05-18

**Authors:** Xuhui Li

**Affiliations:** Engineering Economics Department, Henan Finance University, Zhengzhou 451464, Henan, China

## Abstract

Under the background of the rapid progress of machine learning (ML) and information technology, the traditional classroom model is gradually replaced by the self-media classroom. This thesis aims to solve the problems of understanding abstract content and limited teaching in practical teaching. Based on the ideological and political integration teaching of building architecture, the online classroom design principle reflects the classroom optimization and design principle of building architecture from the perspective of ML. The data advantage is utilized, and the classroom application model is established using the deep learning algorithm through information input. The scene of field survey and building construction is presented from the perspective of mechanization. The simulated results are displayed in the classroom through online teaching combined with ideological education and political teaching mode. The research shows that ML combined with online classroom design breaks through the book face-to-face teaching mode of the traditional classroom through the dynamic demonstration of actual construction, the virtual building structure, and the innovative design of building material entity. It stimulates students' interest in architecture courses, improves the overall learning efficiency, and promotes the ideological and political integration of building architecture courses. Besides, it is conducive to cultivating comprehensive architectural talents in the new era.

## 1. Introduction

With the rapid progress of the global architecture field, multiple schools offer architecture majors, which is essentially a part of engineering education. Keywords in engineering education include engineering ability, job application, practicality, and cooperation. Online learning has gradually become a necessary educational carrier in the age of machine learning (ML). Online education has the advantages of course coverage, ready to accept modification, diversified learning methods, and real-time interaction, which is a powerful tool of present education.

Due to the particularity of the current situation, many schools have added ideological and political elements in the classroom in response to the state's call to cultivate strategic talents. It can actively guide students to focus on courses and majors and form an overall ideological perception in their future work. Steele et al. [1] explored the influencing factors of information placement within the framework of the online classroom. The sample population includes students in the first-year course sequence of a major online college. Qualitative data results show that students' preference is to receive information from multiple access points and sources within the online classroom architecture. The students also express the hope to convey information through technologies such as e-mail and SMS. Fleischmann [2] used blended learning to reshape the architectural design classroom and compared it with one-to-one traditional design teaching activities. The results of communication and feedback show that following the flipped classroom mode, video lectures, software tutorials, and other reading materials are provided online through the learning management system. The effective integration of ideological and political elements and the traditional classroom has become an innovation in the current teaching process. This research shows that many schools face the following problems when integrating ideological and political elements into the classroom. Students' learning objectives conflict with teachers' teaching objectives, and students' needs conflict with the development needs of the current era. Due to the limited class time, it is difficult for teachers to combine current politics with ideological and political elements in the teaching process, so they continue to use the previous traditional teaching mode.

The effective combination and application of ML online teaching and ideological and political elements have been explored to design the architecture of online teaching. By breaking the conventional book face-to-face teaching mode, this thesis aims to use the advantages of the current internet and combine ML algorithms to carry out on-site simulation calculations of the relevant curriculum contents of architecture specialty. The construction industry's relevant drawings and actual on-site operation processes are virtual drills in the online network through virtual reality. This thesis aims to solve the gap between different students' learning focus in the teaching process. The research has improved their ability to deal with problems in the actual work process in the future. In the research process, it is necessary to solve the problem of two-way understanding of each other's needs between students and teachers to further improve the efficiency of classroom learning.

## 2. Materials and Methods

### 2.1. ML

The ML theory includes artificial intelligence (AI), ML, and deep learning (DL). AI covers ML, DL, and reinforcement learning. ML is a method to realize AI and the core of AI, involving multidisciplinary knowledge [3]. In a word, it is the way to realize AI. Data simulation and prediction are carried out through the line of sight of ML algorithms to realize AI technology development [4].  Figure 1 is a DL framework.

Figure 1 reveals that after the calculation of the input layer and hidden layer, DL uniformly processes and outputs the data. The output data are the text after weight reduction to facilitate the next operation and application. The online design of architecture course uses the characteristics of the DL algorithm to simulate and calculate the entity operation data, and obtain the language that the computer can recognize from the output layer for the next simulation and calculation. Then, the machine algorithm is used to predict the text of the data.  Figure 2 is the running flow of the machine algorithm.

Figure 2 reveals that after the data of deep operation are input, the relevant algorithms are used to classify the data, and then, the data nodes and branches are run.  Figure 3 shows the differences and associations among DL, machine algorithms, and AI.

Figure 3 shows that ML relies on DL for algorithm implementation. The data are analyzed and summarized through the algorithm operation, and the simulated data form a unique machine algorithm. AI technology can be synthesized after processing. The evolution of building architecture starts from the most primitive hand measurement and the drawing design to the graphic design in computer-aided design (CAD) drawing in the development of computer technology and to ML, three-dimensional (3D) vertical drawing design under AI, and building information modeling (BIM) technology in recent years. All of these reflect the development of ML technology, which makes the subject classroom in the field of building architecture more and more accurate and effective. Meanwhile, the combination of ideological and political education promotes the healthy development of building architecture, and it is conducive to the cultivation of contemporary strategic talents. Among them, the core of BIM is to provide this model with a complete construction engineering information base consistent with the actual situation by establishing a virtual 3D model of construction engineering and using digital technology. The information base contains geometric information, professional attributes, and state information describing building components, and state information of noncomponent objects (such as space and motion behavior). With the help of this 3D model containing construction engineering information, the degree of information integration of construction engineering is greatly improved to provide a platform for engineering information exchange and sharing for the stakeholders of construction engineering projects.  Figure 4 shows the specific content of the development of building architecture.

### 2.2. ML Algorithm

The ML algorithms can be divided into supervised learning and unsupervised learning.  Figure 5 shows the specific content of the ML algorithm. Supervised learning can be used for the dataset of specific attributes when other data have no labels. The ML training results are artificially specified during the algorithm model training, and the algorithm model will automatically adjust the internal parameters [5]. Unsupervised learning is used in datasets without labels to determine the potential relationship between data and automatically realize data association with national algorithm models [6].

There are various ML algorithms, among which the computational methods of supervised learning are more widely used.

Supervised learning includes linear regression, logistic regression, decision tree, random forest, Naive Bayesian classification, K-nearest neighbor algorithm, ordinary least squares, support-vector machine, and integration method [7].

Unsupervised learning includes clustering algorithm, principal component analysis, singular value decomposition, and independent component analysis [8]. Unsupervised learning is applicable to datasets without labels to find out the potential relationship between data and automatically realize data association with national algorithm models.

Figure 5 presents that the algorithm model is divided into two categories, and supervised learning has a broader scope of application. The operation of this thesis is based on the implementation of Apriori (association rule algorithm) and frequent pattern (FP) growth algorithms in the supervised algorithm. The specific algorithm operation is as follows.

The Apriori is a commonly used algorithm in association analysis to mine frequent itemsets [9]. It is an algorithm to mine association rules through frequent itemsets. The algorithm can find frequent itemsets and mine association rules between items. Support and confidence are used to quantify frequent itemsets and association rules. Its core idea is to mine frequent itemsets through two stages: candidate set generation and downward closure test and detection of plots [10, 11]. The most common improved algorithm is the AprioriTid algorithm. The main difference between this improved algorithm and the original algorithm is that the update method of the dataset is different. When the amount of data is large, the new dataset obtained by using the improved algorithm is much smaller than the original dataset, which saves a lot of time during traversal. The FP growth algorithm is faster than the Apriori algorithm. It is built based on Apriori, but some different technologies are used to complete the same task. Unlike the “generation test” of the Apriori algorithm, the task here is to store the dataset in a specific structure called the FP tree and find frequent itemsets or frequent item pairs, that is, the set FP tree of element items that often simultaneously appear. This approach makes the execution speed of the algorithm faster than Apriori, and the performance is usually better than two orders of magnitude [12, 13]. Its operation steps are as follows:

**Step 1 .**

It is to judge whether the itemset belongs to a frequent set. If not, the contained itemset must not be a frequent set.

**Step 2 .**

If the judged item set is a frequent set, any nonempty subset in it is also a frequent set. At this time, Apriori needs to repeatedly scan the table from the first item to remove the infrequent itemsets, label the relevant infrequent itemsets, and distinguish them with computer language. Set *L* is obtained after deletion. All elements in *L* are freely combined to generate a new set as C. Set C is rescanned to remove infrequent items, and the above steps are repeated [14]. It is assumed that there are the following elements in the field construction scenario, as shown in Table 1 below.

Table 1 shows that after algorithm analysis and removing the infrequent sets from the element sets that may be used in schools, the Logistic regression algorithm is used to run data processing.

The expression of the Logistic function reads the following:

(1) $$\begin{array}{c} h_{\theta }\left(x\right)=g\left(\theta^{T}x\right) \end{array}$$

(2) $$\begin{array}{c} g\left(z\right)=\frac{1}{1+e^{-z}}. \end{array}$$

In the classification prediction function *h*_*θ*_(*x*), vector *x* is known (*x* is object data with the unknown class number), while vector *θ* is unknown, that is, the problem of finding the classification function is transformed into finding the vector *θ*. *θ*^*T*^ is a transpose of vector *θ* (*θ*^0^, *θ*^1^,… , *θ*^*n*^). In vector *X*(*X*^0^, *X*^1^,… , *X*^*n*^), *n* − 1 is the dimension of the data, *X*_0_ = 1. Function derivation is performed according to the original function. *e*^−*z*^ refers to the value corresponding to the exponential function with sample number *z*, and the derivative function g' (*z*) is obtained as follows:

(3) $$\begin{array}{c} g{}^{\prime }\left(z\right)=\frac{d}{dz}\frac{1}{1+e^{-z}}\\ =\frac{1}{{\left(1+e^{-z}\right)}^{2}}\left(e^{-z}\right)\\ =\frac{1}{\left(1+e^{-z}\right)}\cdot \left(1-\frac{1}{\left(1+e^{-z}\right)}\right)\\ =g\left(z\right)\left(1-g\left(z\right)\right). \end{array}$$

For the derivative function *g*′(*z*), in the case of two classifications, *e*^−*z*^ refers to the value corresponding to the exponential function with the sample number of *z*. Function outputs 0 or 1.  Figure 6 presents the final scanning results when removing infrequent sets is not carried out during the operation and the data are directly run without algorithm analysis and scanning.

Figure 6 shows that when infrequent sets are not removed, the algorithm arranges all datasets without dominant differences and the optimization process. The Logistic regression method is mainly to learn the maximum likelihood estimation, so the posterior probability of a single sample is as follows [15]:

(4) $$\begin{array}{c} p\left(y|x;\theta \right)={\left(h_{\theta }\left(x\right)\right)}^{y}{\left(1-h_{\theta }\left(x\right)\right)}^{1-y}, \end{array}$$

*p*(*y|x*; *θ*) represents the probability value of the function when *x* tends to *θ*, and also the probability of category *y* = 1 when *X_i_* is determined. After the probability value of the whole sample is obtained, the posterior probability *L*(*θ*) of the sample is as follows [16]:

(5) $$\begin{array}{c} L\left(\theta \right)=p\left(\overset{⟶}{y}X;\theta \right)\\ =\prod_{i=1}^{m}{\left(h_{\theta }\left(x^{\left(i\right)}\right)\right)}^{y^{\left(i\right)}}{\left(1-h_{\theta }\left(x^{\left(i\right)}\right)\right)}^{1-y^{\left(i\right)}}. \end{array}$$

*L*(*θ*) is a linear probability calculation. It is the probability of category *y* = 0 when the independent variable value *X_i_* is determined. When *y* = 1 and *y* = 0, the probability calculation is as follows:

(6) $$\begin{array}{c} P\left(y=1|x;\theta \right)=h_{\theta }\left(x\right),\\ P\left(y=0|x;\theta \right)=1-h_{\theta }\left(x\right). \end{array}$$

Then, the likelihood function with the number of samples *m* is *L*(*θ*). The likelihood function is changed by logarithmic form, and further simplification is as follows: [17]:

(7) $$\begin{array}{c} \ell \left(\theta \right)=\log\;L\left(\theta \right)\\ =\sum_{i=1}^{m}y^{\left(i\right)}\log\;h\left(x^{\left(i\right)}\right)+\left(1-y^{\left(i\right)}\right)\log\left(1-h\left(x^{\left(i\right)}\right)\right). \end{array}$$

The value of the maximum likelihood function is the required vector *θ*. *L*(*θ*) represents the linear probability. With the change in the value of the independent variables *X^i^* and *Y^i^*, the classification prediction function *h*_*θ*_(*x*) is the value from equation 1, and log is a logarithmic function. If the infrequent sets are removed in each step, the possible infrequent itemsets are represented by shaded parts, as shown in Figure 7.

In Figure 7, the infrequent sets are removed from the scanning results and represented by the shadow. The ML process will further simplify the data and reduce the repetition of operations. Based on this, the online design elements of ideology and politics are evaluated, and the next operation is carried out after removing the repeated set.

The FP growth is an efficient frequent item mining method. Its calculus needs two steps. The first step is to scan to obtain the frequency of the current item, remove the items that do not meet the support requirements, and sort the remaining items [18]. The second step is to build the tree model by scanning and conducting data mining on frequent pattern tree (FP tree) [19]. The algorithm used in data mining is the Iterative Dichotomiser 3 (ID3) decision tree algorithm. It is to select the division characteristics according to the information gain and then recursively construct the decision tree for data collection and processing. Massive candidate datasets are generated by collecting the curriculum design elements of ideological and political education in colleges.  Table 2 shows the data elements after analysis and processing.

As described in Table 2, the elements are represented by data classification and classified by different fulcrums. The weight value is given to the data. After the above Apriori algorithm distinguishes common materials, the FP tree of the corresponding materials in Figure 8 is generated.

In Figure 8, the most frequently used ones are listed in the first column, which is arranged downward by nodes to find the cardinality of qualified patterns, propose frequent sets, and further filter and simplify the data.

The pattern base suitable for the single item *P* with the lowest frequency is found first. Similarly, the FP tree construction method is used to construct the FP tree under the pattern base, and the frequent set of P is found on this tree [20]. Then, frequent itemsets are sequentially mined from the conditional pattern bases of p, m, b, a, c, and f.

### 2.3. ML Algorithm in the Field of Building Architecture

Building construction consists of planning, design, construction, operation, and maintenance stages. In each stage, a large amount of data will appear during operation. In the construction supervision and operation and maintenance control stage, the existing data flow can be displayed to students in electronic form during online teaching. There are data streams sorted by time series to facilitate sorting and use [21]. The ML algorithm is usually used in the building information model (BIM)-based design stage. It can also be applied to environmental monitoring, labor safety, and other scenes in construction [22]. ML is being applied worldwide, which significantly improves the safety of building construction [23]. There are three main reasons for the rapid development of ML in architectural security. The cloud and mobile internet technology are adopted in engineering management; data source acquisition during construction is explosive; and ML and DL technology are rapidly developing. The research and development personnel of ML, especially in the branch of DL, have made a breakthrough. Recent progress shows that the system can translate high-performance speech algorithms in real time and monitor the surrounding environment in real time, as shown in Figure 9 below.

Figure 9 reveals that the DL network structure arranges the data into logical data for later output through complex operations.

### 2.4. Ideological and Political Design of Building Architecture Course

Data are explosively growing with the use of mobile internet technology on construction sites. Relevant on-site staff use the data for verification and review, conduct safety observation, and upload the records to the system for verification. According to this situation, teachers should integrate building architecture and ideological and political design into the classroom to improve the students' real feelings. They can show students the scene of site work through VR for interactive teaching and adopt computer algorithms for field simulation exercises to cultivate students' real sense of experience and improve classroom efficiency. Learning the curriculum design of building architecture can enhance human happiness and a sense of belonging. It can further help teachers timely master students' learning situations and dynamics to improve the classroom's accuracy [24].  Figure 10 is a specific display.

Figure 10 shows the influence of the course design of building architecture on the students and the principle of the course setting. It presents the students with a more intuitive class experience and feeling from the computer perspective.

Besides, when massive building data exist in the plane, people often ignore their laws and connections. However, when the computer is used to sort out the data and present the 3D image, the impact experience for the students is more intuitive. It can promote their enthusiasm and learning motivation for building architecture and stimulate the students' ability of hands-on operation [25], as shown in Figure 11.

In Figure 11, knowledge in the classroom can be displayed in the form of a physical map from the perspective of computer, which can better stimulate students' motivation and enthusiasm in class. The architecture course is systematically simulated and designed through the above methods. After distinguishing common materials with the Apriori algorithm, the FP tree is generated as follows. The Logistic regression algorithm shows the generated result data and relevant data analysis in the result part. The development of cloud technology also makes it possible to aggregate data into one location for analysis. Multiple projects and buildings need to be analyzed in combination with the local environment and terrain, which can be achieved by developing computer and cloud technology [26]. Online teaching is adopted to clearly show the steps of this process to students. In the future, it can also effectively improve students' hands-on operation ability in practical operations [27]. BIM technology and AI are used in combination to work, as shown in Figure 12 below.

Figure 12 reveals that BIM and AI are combined to conduct unified data-based learning and sorting of building architecture, and the teaching of traditional building architecture is based on paper books. Students cannot empathize, so there is an inefficient or even ineffective classroom. The building architecture under ML removes the traditional teaching concept and integrates the calculation and operation entity effect to show the charm of building architecture. In the overall teaching process, the use of computers in ideological and political teaching is more effective and conducive to students. It improves the students' practical ability while changing the traditional teaching concept and optimizing the teaching concept of ideological and political education. In addition to the full understanding of architectural design, the teaching goal should also include understanding the principles and methods of architectural design, using computer technology, and drawing construction ability. On this basis, ideological and political education elements are integrated, and college students in the new era are cultivated. Meanwhile, the perspective of ML improves students' learning enthusiasm and optimizes the classroom order.

## 3. Results and Discussion

### 3.1. Accuracy Analysis of Online Teaching Design Results and Simulation Results

According to the research materials, if the student group is fixed, the error simulation analysis of the online classroom design of architecture course is carried out using the Apriori algorithm, FP tree, and Logistic regression algorithm, as shown in Figure 13 below.

In Figure 13, in the two-hour online course, the overall display error of the Apriori algorithm is relatively small and the stability is high. The relationship between data loading and network operation in the first 20 minutes leads to an increase in error rate. After the stable operation in the later stage, the overall classroom effect error is the smallest. The error of the Logistic algorithm in the main course is relatively high, and there are certain errors in entity operation and theory. The FP tree is relatively stable in the operation process, the error range is also relatively low, and there are relatively small errors in the accuracy and selection indicators of the tree building model.  Figure 14 displays the measurement results of the overall classroom operation accuracy.

Figure 14 shows that the running accuracy of the whole algorithm is maintained between 0 and 1. The calculation accuracy of the Apriori algorithm fluctuates relatively large, because it effectively uses the real-time changing data for site monitoring and simulation operation in operation. Hence, there is a significant accuracy difference in the operation process. The accuracy of the Logistic algorithm is relatively high in the overall operation process, and the operation process is also very smooth. Therefore, there will be no classroom delay or inaccuracy in the operation process. Physical simulation is carried out based on the running process of the three algorithms. The simulation data are further optimized according to the field experimental objects.  Figure 15 displays the specific performance.

Figure 15 shows that after using the optimization algorithm to train the overall operation process, the overall optimal solution of the different number of field experimental objects can be obtained (*A*). Moreover, the running time and running quantity tend to be stable (B). When the sample data are running, the difference between the average and test errors between the algorithms is between 0.1 and 0.35 (C), significantly reducing the error range. Based on the online model proposed, the DL model of sample training is adopted to analyze the effect of students' learning in the online classroom and the excellence of ideological and political integration into the classroom. It can help teachers further effectively evaluate students' abilities and carry out the next teaching design and preparation.

This thesis shows that the online teaching design of ideological and political education of housing architecture from the perspective of ML is a new classroom experience for contemporary students. It also promotes the effective integration of professional education and online ideological and political education and promotes the formation of an efficient talent training strategy. Meanwhile, the combination of ML perspective and real ground engineering is conducive to cultivating students' pragmatic and rigorous discipline thinking while looking for ideological and political elements. The building architecture is not just talking on paper but by comparing various online computing models and field VR. Besides, it is combined with the current hot spots to adapt to the rapidly changing data era. In this way, teachers can timely adjust the class content and scheme. The building architecture is effectively combined with ML by integrating with the ideological and political background.

### 3.2. Results and Discussion

Through ML-related technology's architecture, by revealing the data processing of the input layer and hidden layer in the network model, the DL algorithm is used to realize the graphical design of architectural design drawings. The frequent item dataset is mined and processed by ML unsupervised learning algorithm, and the error simulation analysis of online classroom design of architecture course is carried out by using the Apriori, FP tree, and Logistic regression algorithms. The results show that the overall display error of the Apriori algorithm is relatively small, and its stability is high. FP tree is relatively stable during operation, and the error range is relatively small. These results are consistent with the expected research results. For example, scholar Susilo [28] studied the application of the Apriori algorithm in processing the supermarket sale transaction data, with the development of the mini-market as an example. The results show that using the Apriori algorithm in the process of commodity sale data processing can improve data processing efficiency. Edadama et al. [11] used the Apriori algorithm to realize glass sale data mining. The research shows that the ability of the system to collect and process data is improved by using the Apriori algorithm. Narvekar et al. [29] studied the optimization algorithm of association rule mining based on the FP tree and found hidden or desired patterns from massive data through association rule mining. The research greatly reduces the time efficiency of the algorithm. To sum up, the research on ML unsupervised learning algorithms proves the effectiveness of the Apriori algorithm, and the research results here are also consistent with the results of these studies.

## 4. Conclusions

Based on the DL algorithm of ML, the relevant theoretical basis in building architecture, online curriculum design, and ideological and political ideas are analyzed. The online course system based on the DL algorithm is constructed and integrated with ideological and political elements for classroom practice. By integrating ideological and political elements into the classroom teaching of building architecture, ML algorithm and VR online form are used to show the text in the textbook to the classroom in the form of the real scene online. Then, students can feel the scene in practical work and learn to deal with practical problems. In addition, the optimization of the DL algorithm ensures the stability and more accurate dissemination accuracy of the online classroom, reduces the information omission and loss caused by the data transmission process, and obtains the optimal solution of data simulation in the fieldwork scene. Using the proposed DL algorithm in the online course design practice of building architecture can help colleges improve the practice quality of building architecture. It puts forward new ideas for the design of contemporary building architecture teaching courses and points out a new direction for training new talents in building architecture. The research innovation is to give full play to the advantages of the online classroom from mechanization and realize the integration design of discipline and professional theoretical knowledge and ideological and political design. This concept meets the needs of the current era, helps to cultivate high-end engineering and technical talents, and promotes the professional education value of disciplines with Chinese characteristics. The research deficiency is that it cannot be popularized and used in a short time because of the high demand for science and technology. Future research will focus on simplifying the popularization and operation requirements of the algorithm to promote further development and application.

## Figures and Tables

**Figure 1:** DL architecture.

**Figure 2:** Flow of machine operation.

**Figure 3:** Relationship between AI, ML, and DL.

**Figure 4:** Development history of building architecture.

**Figure 5:** ML algorithm.

**Figure 6:** Optimization steps without removing infrequent sets.

**Figure 7:** Algorithm steps for removing frequent sets.

**Figure 8:** Structure of FP tree.

**Figure 9:** Operation system of DL.

**Figure 10:** Function of course design of building architecture.

**Figure 11:** Display of ML effect.

**Figure 12:** BIM and AI cooperation operation diagram.

**Figure 13:** Online teaching design error.

**Figure 14:** Accuracy of architectural ideological and political online teaching design.

**Figure 15:** Simulation results of teaching effect ((a) the running time of the algorithm to obtain the optimal solution, (b) the running steps and running time of the algorithm, and (c) the error value in the running process of the algorithm).

**Table 1:** List of element items.

Example	Transaction number	Items
1	0	f, a, c, d, g, I, m, p
2	1	a, b, c, f, I, m, o
3	2	b, f, h, j, o
4	3	b, c, k, s, p

**Table 2:** Data mining and branch processing.

TID	Items	(Ordered) frequent items
100	f, a, c, d, g, I, m, p	f, c, a, m, p
200	a, b, c, f, I, m, o	f, c, a, m, b
300	b, f, h, j, o	f, b
400	b, c, k, s, p	c, b, p
500	a, f, c, e, l, p, m, n	f, c, a, m, p

## Data Availability

The data used to support the findings of this study are available from the corresponding author upon request.
